# Acute airway obstruction requiring nasotracheal intubation following hypoglossal neuromonitoring: a case report

**DOI:** 10.1186/s12871-023-02115-y

**Published:** 2023-05-03

**Authors:** Jaspal Singh Bassi, Frank Hsu, Lilit Mnatsakanyan, Govind R. Rajan

**Affiliations:** 1 University of California Irvine School of Medicine, 836 Health Sciences Road, Irvine, CA 92697 USA; 2 Department of Neurological Surgery, University of California Irvine Medical Center, 101 The City Drive South, Orange, CA 92868 USA; 3 Department of Neurology, University of California Irvine Medical Center, 101 The City Drive South, Orange, CA 92868 USA; 4 Department of Anesthesiology and Perioperative Care, University of California Irvine Medical Center, 101 The City Drive South, Orange, CA 92868 USA

**Keywords:** Neurophysiological monitoring, Hypoglossal, Nerve, Lingual swelling, Nasotracheal intubation

## Abstract

**Background:**

Intraoperative neurophysiological monitoring (IONM) is utilized for both the localization of critical structures and for real time detection and prevention of intraoperative neurological injury. Use of IONM to monitor the hypoglossal nerve is performed during neurosurgical, otolaryngological, and vascular procedures to improve surgical outcomes. There is a paucity of literature describing potential complications of IONM of the hypoglossal nerve, especially with respect to airway compromise. Here we present our findings regarding a case of acute airway obstruction following hypoglossal nerve monitoring.

**Case Presentation:**

A 54-year-old male was admitted for left far-lateral craniotomy and microsurgical clipping of a left posterior inferior cerebellar artery (PICA) aneurysm. Following induction and intubation but prior to the procedure start, the patient was placed in the ¾ prone position with the left side up and his neck was flexed approximately 10 degrees. He then underwent placement of subdermal needle electrodes into the facial muscles, trapezius muscles, soft palate, and tongue for IONM. The procedure lasted 523 minutes and was completed without complication. However, approximately one hour after emergence from general anesthesia, the patient experienced progressive difficulty breathing secondary to severe lingual swelling. He required emergent placement of a nasotracheal tube guided by a fiberoptic bronchoscope. He remained intubated for 3 days and was treated with dexamethasone, after which the swelling resolved, and the patient was successfully extubated.

**Conclusions:**

Acute lingual edema is a potentially life-threatening phenomenon that can lead to rapid airway compromise. Generally, causes of acute lingual swelling include hemorrhage, edema, infarction, and infection. In the case described above, we suspect traumatic injury to the tongue’s vascular supply caused a deep tissue hematoma leading to postoperative acute lingual swelling and airway obstruction. With the widespread use of IONM, it becomes essential for providers to be aware that perioperative airway compromise is a potentially life-threatening complication, especially with respect to monitoring of the hypoglossal nerve. Awake fiberoptic nasotracheal intubation can successfully be employed to establish an emergency airway in such situations.

## Background

Intraoperative neurophysiological monitoring (IONM) is a common method used to monitor the neurological status of patients under general anesthesia during neurological surgery. It allows for both the localization of critical structures and for real time detection and prevention of intraoperative neurological injury [1, 2]. Use of IONM to monitor the hypoglossal nerve is often performed to improve surgical outcomes and minimize postoperative injury in those receiving skull base surgery [3]. Outside of skull base procedures, hypoglossal nerve monitoring is conducted in a variety of otolaryngological surgeries, carotid endarterectomy, and even in the treatment of obstructive sleep apnea [4–6]. Monitoring is often conducted by placing electrodes percutaneously in the lateral aspect of the tongue [3, 5]. While generally considered safe, there is a paucity of literature describing potential complications of IONM of the hypoglossal nerve, especially with respect to airway compromise. In this case report, we discuss a unique case of lingual swelling following hypoglossal nerve monitoring and the management of this complication.

## Case report

A 54-year-old male was admitted to the hospital for left far-lateral craniotomy and microsurgical clipping of a left posterior inferior cerebellar artery (PICA) aneurysm. He initially presented with vertigo, headache, and intermittent blurry vision. He subsequently underwent a computed tomography scan of his head followed by computed tomography angiogram which revealed an unruptured left PICA fusiform aneurysm measuring 3.9 mm x 3.7 mm. x 3.7 mm.

The patient had a history of well-controlled hypertension, was able to participate in 7–10 metabolic equivalents of task, had a body mass index (BMI) of 28.1 kg/m^2^, and had an American Society of Anesthesiology (ASA) score of 2. He had no known adverse reactions to anesthetic agents in the past. In the operating room, the patient was induced with fentanyl, lidocaine, propofol and succinylcholine. Succinylcholine was used as a paralytic because its short half-life would enable it to be quickly metabolized to allow for IONM. Orotracheal intubation was successfully performed with a 7.5 mm endotracheal tube and a soft bite block was placed. The patient was maintained under total intravenous anesthesia using propofol and remifentanil and was mechanically ventilated. Following induction and intubation but prior to the procedure start, the patient was placed in the ¾ prone position with the left side up and his head affixed in a three-point head holder. His neck was flexed approximately 10 degrees. He then underwent placement of subdermal needle electrodes for IONM. Electrodes were placed into the left frontalis, orbicularis oculi, orbicularis oris, and mentalis muscles for electromyography (EMG) of the facial nerve. Additional electrodes were placed in the left trapezius muscles for EMG of the accessory nerve, soft palate for EMG of the glossopharyngeal nerve, and tongue for EMG of the hypoglossal nerve. A single 12 mm long electrode was inserted at an approximately 45-degree angle on the left lateral side of the tongue. Additional IONM included somatosensory evoked potentials (SSEP) of the median nerve and brainstem auditory evoked potentials. The surgery lasted approximately 523 minutes, was completed without complication, and IONM demonstrated no apparent injury to the neurological structures.

The patient was extubated successfully and without any evidence of lingual swelling. Approximately 30 minutes later however, the patient was noted to have mild, non-obstructing lingual swelling in the post anesthesia care unit. At that time, he was able to maintain his airway and swallow secretions. On physical exam, there was mild excoriation noted on the left side of the tongue in the area of electrode placement without any obvious trauma, laceration, or bleeding. Approximately one hour later, however, upon transfer to the Neuroscience Intensive Care Unit, the patient experienced progressive difficulty breathing secondary to massive lingual edema (Fig. 1). Stridor was not appreciated and there was no swelling noted in the patient’s submandibular or neck area. The patient’s airway was obstructed, and he required emergent placement of a nasotracheal tube. An atomizer was used to anesthetize the right naris, pharynx, vocal cords, and trachea with 7.0-cubic centimeters of 4% lidocaine. A 7.0-millimeter nasotracheal tube was placed in the right naris and was guided without complication into the trachea using a fiberoptic bronchoscope. Correct placement of the nasotracheal tube was confirmed by visualizing the tube above the carina.

**Fig. 1:** Acute post-operative lingual swelling Acute lingual edema seen upon transfer to the ICU, prior to nasogastric intubation. Photo taken approximately 1 hour following extubation

Following emergent stabilization, the patient was unable to move the tongue or swallow secretions due to the massive lingual edema. The patient was seen by otolaryngology and fiberoptic examination of the oropharynx revealed the tongue completely occluding the extent of the oropharynx without any visible laceration or bleeding from the tongue. The scope was unable to be advanced to visualize the posterior tongue or vocal cords. He required treatment with eight milligrams of dexamethasone every six hours. Over the following days, the patient was able to regain movement of his tongue and better manage his secretions as the edema decreased. On post-operative day 3, he was successfully extubated, and the dexamethasone dose was tapered and eventually discontinued. No further treatment of the lingual edema was required, and the patient otherwise did well post-operatively.

## Discussion

Acute lingual swelling is a potentially life-threatening phenomenon that can lead to rapid airway compromise. Generally, causes of acute lingual swelling include hemorrhage, edema, infarction, and infection [7]. Post operative macroglossia is a known complication of neurological procedures, especially among craniotomies conducted in the sitting position [8, 9]. In these cases, extreme neck flexion likely resulted in impaired venous drainage of the tongue leading to edema. In our case, the patient was positioned ¾ prone, and the head was flexed at approximately 10 degrees. It is possible this amount of flexion could have resulted in partial local venous compression or lymphatic obstruction. Additionally, if arterial or venous flow was partially obstructed during the prolonged procedure, reperfusion injury following the procedure likely contributed to this patient’s presentation.

Another likely etiology in this case is hematoma formation caused by traumatic arterial injury secondary to electrode placement. Evaluation by otolaryngology revealed that while there was no surface hematoma that could be drained, the needle electrode may have caused arterial injury within the deep tissue causing post-operative lingual swelling once removed. The tongue is a relatively well vascularized structure, receiving blood supply from the lingual artery and its branches. Cases of penetrating injury to the tongue resulting in disruption of the lingual artery causing edema and airway compromise have previously been described [10, 11]. Several studies have also identified anticoagulation therapy as a risk factor for airway obstruction due to the formation of sublingual hematomas [12, 13]. Interestingly, however, our patient experienced this complication without receiving any anticoagulation. To our knowledge, this is the first described case of lingual edema with placement of electrodes used for IONM of the hypoglossal nerve as a likely contributor.

Other potential but less likely causes include traumatic injury to the tongue secondary to IONM. It has been well documented that transcranial motor evoked potentials (Tc-MEPs) can result in tongue biting injuries that can lead to lingual swelling [14]. This is less likely in our case as this patient underwent only EMG of the hypoglossal nerve and there were obvious lacerations visible on the tongue post-operatively. Another potential cause could have been edema secondary to hereditary angioedema or an allergic reaction [7]. However, this patient had no personal or family history of hereditary angioedema and his only antihypertensive medication was daily amlodipine. His only allergies were to iodinated radiocontrast agents and he did not have any reaction to anesthetics used in his prior surgery. The medications administered towards the conclusion of the case included dexamethasone, ondansetron, fentanyl, and cefazolin. There was no rash, change in vital signs, swelling outside the area of the tongue, or other symptom to suggest allergic reaction as a cause of his lingual swelling.

The case discussed here highlights the importance of caution when employing neurophysiological monitoring of the hypoglossal nerve. Use of such monitoring can provide valuable input to surgeons when performing skull base surgeries. In these cases, it is vital for anesthesiologists to be aware that both the amount of neck flexion and injury caused by insertion of a needle electrode can lead to acute lingual edema resulting in airway obstruction. To prevent such complications, we recommend avoiding the sitting position for craniotomies and the use of extreme neck flexion to prevent vascular and lymphatic obstruction. To avoid pressure injury secondary to endotracheal tube placement, nasotracheal intubation may be employed if the patient has no contraindications. Additionally, caution should be noted when placing needle electrodes used for IONM. Because of the vascularity of the tongue, it is difficult to describe optimal placement of the electrode to avoid vascular injury. However, use of a short and thin electrode can help mitigate this risk. When such emergency does occur, maintenance of the patient’s airway is critical. Orotracheal intubation may be difficult or impossible due to severe macroglossia. We recommend nasotracheal intubation with the assistance of a fiberoptic bronchoscope. This allows for visualization of the airway and accurate placement of the tube within the trachea. This technique has been utilized by other studies requiring placement of an emergency airway in patients suffering from acute macroglossia [15, 16]. Urgent cricothyroidotomy should be reserved as a last option but may be required in the setting of severe airway obstruction, especially if complicated by laryngeal edema [9]. In this case the lingual edema was successfully treated with supportive care and corticosteroids to decrease the inflammatory response. In cases with more severe injury and obvious hematoma formation, angiography and embolization can be considered [17].

## Conclusion

With the widespread use of IONM, it becomes essential for providers to be aware that monitoring of the hypoglossal nerve can contribute to and exacerbate acute lingual swelling leading to perioperative airway compromise. In such cases, awake fiberoptic nasotracheal intubation can successfully be employed to establish an emergency airway.

## Data Availability

Not applicable, as this study is descriptive in nature and no datasets were generated for this study. Case-relevant details are included in the manuscript body.

## Abbreviations

IONM: Intraoperative neurophysiological monitoring
PICA: Posterior inferior cerebellar artery
Mm: Millimeter
BMI: Body mass index
ASA: American Society of Anesthesiology
EMG: Electromyography
SSEP: Somatosensory evoked potentials
Tc-MEP: Transcranial motor evoked potentials
